# Effect of Enhanced Recovery after Surgery (ERAS) Concept and Cluster Nursing on Psychological State and Pain of Oral Outpatients Undergoing Root Canal Therapy

**DOI:** 10.1155/2022/4868569

**Published:** 2022-09-10

**Authors:** Bei Liu, Mao Xiong, Feng Liu, Wenyu Chen, Shumei Jiang, Meixiang Qu, Lixiang Mao, Genyun Yi, Xiongwei Liu, Yuehui Wang

**Affiliations:** ^1^Department of Stomatology, Hunan Provincial People's Hospital (The First Affiliated Hospital of Hunan Normal University, Changsha City, Hunan Province 410005, China; ^2^Outpatient Office, Hunan Provincial People's Hospital (The First Affiliated Hospital of Hunan Normal University, Changsha City, Hunan Province 410005, China

## Abstract

**Objective:**

The effect of the concept of enhanced recovery after surgery (ERAS) and pain of patients undergoing root canal therapy in oral clinic.

**Methods:**

200 participants in an oral clinic from March 2020 to March 2022 were enrolled in our study. The control group (*n* = 100) accepted ERAS-based care and the research group (*n* = 100) accepted ERAS concept and cluster nursing. Nursing satisfaction, comfort, self-efficacy, subjective well-being, self-rating anxiety scale (SAS), and self-rating depression scale (SDS) scores were compared.

**Results:**

The research group had 100% satisfaction rate; the control group had 87% satisfaction rate. After nursing, the scores of comforts and self-efficacy of the two groups increased and the scores of comforts and self-efficacy of the research group were higher than those of the control group. After nursing, the scores of subjective well-being of the two groups increased. Furthermore, the higher scores of life satisfaction, interpersonal harmony, and self-efficacy in the research group were found. There was no significant difference in the scores of SAS and SDS between the two groups before nursing (*P* > 0.05), but after nursing, the scores of SAS and SDS in the two groups decreased, and the scores of SAS and SDS in the research group were lower than those in the control group, and there are statistically significant differences between the groups (*P* < 0.05). The scores of visual analogue score (VAS) and numerical rating scale (NRS) following intervention decreased, and there are statistically significant differences between the groups (*P* < 0.05). The less physiological, psychological, social functions, and health self-cognition in the research group were displayed, and there are statistically significant differences between groups (*P* < 0.05).

**Conclusion:**

The adoption of the concept of ERAS and cluster nursing can effectively improve the psychological state and pain score of oral outpatients undergoing root canal therapy, improve comfort and self-efficacy, and enhance subjective well-being and quality of life. ERAS and cluster nursing is of great significance in relieving pain after root canal therapy in the outpatient department, reducing patients' pain and improving patients' quality of life.

## 1. Introduction

Periapical periodontitis is mainly characterized by the absorption of periapical bone tissue, which remains one of the common diseases in oral clinical work, seriously influencing the oral health and quality of life of patients. Oral health is one of the important indicators of human body health. In 1981, the World Health Organization (WHO) defined oral health standards as follows: clean teeth, no caries, no pain, normal gingival color, and no bleeding [1]. Furthermore, pulpitis and periapical periodontitis are the pathological changes of inflammation, suppuration, and necrosis of dental pulp caused by bacterial infection, physical and chemical stimulation, and immune response and even spread to the periapical tissue, causing inflammation and absorption of periapical tissue [2]. Of note, infection control is the core principle for the treatment of pulpitis and periapical periodontitis. Whitehouse supports this view for a long time and regards this view as the basic standard to guide clinical operation [3]. For more than one hundred years, there are two main ways to treat dental pulp disease and periapical disease: thorough debridement and harmless. Root canal therapy is a method developed based on the former as the basic principle. At present, the most ideal treatment for pulpitis and periapical periodontitis is root canal therapy, but in the process of root canal therapy, patients often have a certain degree of pain, intraoperative pain leads to patients being unable to cooperate with the doctor to complete the operation and even interrupts the treatment, and the patients refuse to see a doctor again. This kind of pain and discomfort can lead to anxiety, depression, irritability, and negative rebellious coping style; bad emotional state and coping strategies worsen doctor-patient relationship, reduce patients' trust in doctors, and patients evading treatment [4]. Therefore, the oral health condition is getting worse and worse, the quality of life cannot be guaranteed, and the well-being index of life is greatly reduced [5, 6]. Therefore, the purpose of this study was to investigate the effect of enhanced recovery after surgery (ERAS) concept and cluster nursing on the psychological state and pain of patients undergoing root canal therapy in dental clinics.

## 2. Patients and Methods

### 2.1. Patient Clinical Data

200 patients of root canal therapies in oral clinic from Mar. 2020 to Mar. 2022 were selected.

The inclusive criteria were as follows: (1) patients who needed root canal therapy because of periapical periodontitis, pulpitis, and pulp necrosis (posterior molars), (2) patients had no systemic disease, (3) patients had no abnormal reaction and coping ability in normal life, (4) patients did not take painkillers and antibiotics within 1 month before treatment; and (5) those who volunteered to participate in this study and were able to return on time.

Exclusion criteria are as follows: (1) pregnant and breastfeeding patients; (2) patients whose oral pain could not be relieved due to periodontitis, periodontitis, pericoronitis of wisdom teeth, temporomandibular joint disorder syndrome, etc.; (3) those who could not complete the treatment and return on time as prescribed by the doctor; (4) those with a history of mental illness; (5) history of pain in other parts of the body and history of severe somatic diseases; and (6) inability to describe their feelings clearly and accurately. Seven cases of root canal filling showed that the overfilling was larger than that of 1 mm by X-ray.

### 2.2. Treatment Methods

The control group received routine nursing intervention. Since the control group, the research group used the concept of ERAS and cluster nursing. The designated initiatives were as follows: (1) take head nurse of oral clinic as the group leader and select the backbone nurses of the department as the group member according to the voluntary principle. When there are problems that nurses cannot solve or need to optimize and improve the process in clinical practice, (2) the team leader organized thematic learning to train and assess the team members to ensure the ERAS cluster nursing strategy. At the same time, the head nurse organized for general practice nurses and obtained the recognition and support of other nurses to ensure the homogeneity of nursing measures. (3) Psychological nursing: actively and actively communicate with patients and tighten the distance between nurses and patients. Self-rating anxiety was used to evaluate the negative emotional state of patients and understand the causes of patients' worry and patiently guide them. The use of comfort, empathy, and other ways was analyzed to help patients with negative emotions, to introduce to patients the ideal quality of life of patients after dental root canal therapy, and to help patients to reconstruct their psychological balance. In strengthening health education, we introduce the related problems of postoperative recovery to the patients before the start of root canal therapy and explain the effect of the operation, so that the patients can rest assured. Before treatment, PPT was used to introduce postoperative nursing precautions to patients and to explain the effects of exercise, bath, diet, interpersonal communication and complications on prognosis, so as to let patients choose reasonably according to their own needs, evaluate their self-nursing ability, correct patients' misoperation in time, and continue until patients were discharged from hospital. We explain the postoperative diet and life matters needing attention, teach them how to keep the mouth clean, and enhance the patients' self-confidence. In pain nursing, when root canal therapy is carried out, gentle action is required to reduce stimulation. Patients are encouraged to supplement food properly before changing dressing in order to increase their pain threshold. When changing medicine, pay attention to the guidance of patients, divert their attention, and guide patients to cooperate in order to reduce pain. Adjust the temperature and humidity of oral clinic to improve the comfort of patients.

### 2.3. Evaluation Index

#### 2.3.1. Satisfaction

After consulting the literature and experts' discussion, we designed patients' follow-up satisfaction [7]: Satisfaction rate = (very satisfied + common satisfied)/total number of cases × 100%.

#### 2.3.2. Comfort and Self-Efficacy Scores

In comfort [8], we evaluate the comfort of patients, including treatment comfort, environmental comfort, temperature comfort, and nursing comfort. In self-efficacy, before and after the intervention, the Chinese version of the general self-efficacy scale [9] was used to evaluate the self-efficacy scale.

#### 2.3.3. Subjective Well-Being Score

For subjective well-being, patients were assessed with Oxford well-being questionnaire (revised version) [10] before and after intervention. The scale included life satisfaction, interpersonal harmony, and self-efficacy with a total of 29 items.

#### 2.3.4. SAS and SDS Scoring

(1) Self-rating anxiety scale (SAS), also known as Zung anxiety scale [11], was compiled by W.K. Zung in 1971. According to the results of the Chinese norm, the standard cut-off value of SAS was 50 points, of which 50-59 points were mild anxiety, 60-69 points were moderate anxiety, and more than 69 points were severe anxiety. (2) Self-rating depression scale (SDS). [12] is a self-rating scale with 20 items, which is divided into 4 grades. The prototype is the depression scale compiled by W.K. Zung (1965). 53-62 was mild depression, 63-72 was moderate depression, and over 73 was severe depression.

#### 2.3.5. Pain Score

In patient self-evaluation, the visual analogue score (VAS) [13] was used to evaluate pain. In nurse evaluation, the numerical rating scale (NRS) method [14] is the most common method to evaluate pain intensity. NRS method describes the strongest level of pain as the number 10 and painlessness as 0. If the pain symptoms are mild, between 1 and 3, the patient is mild pain; if the pain symptoms are severe, between 8 and 10, the patient is severe pain; and the pain symptoms between 5 and 7 are moderate pain symptoms.

#### 2.3.6. Quality of Life Scale

The quality of life scale [15] consisted of four subscales with a total of 29 items. The scale was scored by 1-5 grades.

### 2.4. Statistical Analysis

IBM SPSS 24.0 software was applied for statistical analysis. The measurement data were expressed by mean ± standard deviation. The counting data were expressed by frequency or rate. *t*-test was used when measurement data obey normal distribution, and rank sum test was used when it did not obey normal distribution. *χ*^2^ test was used to compare the classified counting data. Repeated measurement data were analyzed by repeated measurement analysis of variance. Main effect test results were used when there was no interaction, and simple effect analysis was carried out when there was interaction. *P* < 0.05 indicated that the difference between groups is statistically significant.

## 3. Results

### 3.1. Comparison of Nursing Satisfaction

The research group had 100% satisfaction rate; the control group had 87% satisfaction rate. The nursing satisfaction in the research group was higher than that in the control group (*P* < 0.05). All results are shown in Figure 1.

### 3.2. Comparison between Comfort and Self-Efficacy

After nursing, the scores of comfort and self-efficacy were upregulated. The larger scores of comforts and self-efficacy were displayed in a studied cohort, and the difference was statistically significant, and there are statistically significant differences between groups (*P* < 0.05). All results are shown in Table 1.

### 3.3. Comparison of Subjective Well-Being Score

The upregulated scores of life satisfaction, interpersonal harmony, and self-efficacy in the research group were shown statistically, and there are statistically significant differences between groups (*P* < 0.05). All results are shown in Table 2.

### 3.4. SAS and SDS Score Comparison

Following care, the scores of SAS and SDS in the two groups reduced, and there are statistically significant differences between groups (*P* < 0.05). The downregulated scores of SAS and SDS in the study cohort were discovered, and there are statistically significant differences between groups (*P* < 0.05). All results are shown in Table 3.

### 3.5. Pain Score Comparison

The scores of VAS and NRS in the two groups decreased following care, and there are statistically significant differences between groups (*P* < 0.05). The lower scores of VAS and NRS in the study were displayed, and there are statistically significant differences between groups (*P* < 0.05). All results are shown in Table 4.

### 3.6. Comparison of Quality of Life Scores

The lower scores of physiological, psychological, social functions, and health self-cognition in the research group were found, and the difference was statistically significant, and there are statistically significant differences between groups (*P* < 0.05). All results are shown in Table 5.

## 4. Discussion

This study was to investigate the effect of enhanced recovery after surgery (ERAS) concept and cluster nursing on the psychological state and pain of patients undergoing root canal therapy in dental clinics. Periapical periodontitis, also known as periapical disease, is a common disease harmful to oral health. Inflammation occurs in periapical tissues, including periapical membrane, periapical cementum, and periapical alveolar bone; most of them are induced by the secondary pathogenesis of pulpitis, that is, infected dental pulp, bacteria, and other substances acting on the periapical tissue through the apical foramen [3]. Poor oral health behavior brings a lot of inconvenience to everyone's life, such as directly affecting masticatory function and also affecting speech, appearance, psychological activities, and even overall health [5]. In addition to dental caries and periodontitis, periapical periodontitis is also one of the most common oral diseases that interfere with oral health. Periapical periodontitis is an inflammatory disease that occurs around the apical tissue. Most of periapical periodontitis are the secondary diseases of dental pulp disease, which is mainly induced by the action of infectious substances in the root canal on the periapical tissue through the apical foramen, so it is also called periapical disease [16]. The range of periapical periodontitis includes inflammation of the periapical periodontal ligament, cementum, and alveolar bone [17]. Periapical periodontitis is one of the common dental hard tissue diseases. The etiology of periapical periodontitis includes not only bacterial factors, that is, infection factors, but also physical factors such as stimulation of chemicals such as phenols and aldehydes and trauma. According to its clinical manifestations and histopathological process, periapical disease can be divided into acute periapical periodontitis and chronic periapical periodontitis. The main symptoms of the former are severe tooth pain, dare not bite, and gingival and facial swelling, affecting the patient's work, study, and life [18]. Periapical inflammation can also spread to the jaw and surrounding tissue, when the resistance is low, which can form jaw osteomyelitis and cellulitis. If it is not treated in time, it may develop into septicemia and life-threatening. The latter is mostly chronic inflammation of periapical tissue promoted by chronic stimulation for a long time; that is, it often brings about different degrees of destruction of apical alveolar bone and occlusal discomfort. If it is not treated in time, it may become the focus of infection and results in diseases of distant organs of the body [19, 20]. In addition to the subjective factors of clinicians, the success rate of root canal therapy is also different, and the recovery time of apical bone defect after root canal treatment is different, which ultimately affects the recovery of tooth function. That is, the more periapical bone tissue damage defect (the larger the periapical transmission shadow on the X-ray film), the more complex the pathological process, the lower the success rate of root canal therapy, and the longer the postoperative recovery time. Therefore, early prevention, early diagnosis, early treatment, and regular follow-up are very indispensable in clinical work [21, 22].

The destruction degree of the apical alveolar bone of the teeth with periapical disease is different, the kinds of bacteria infected are different, the clinical pathological process is different, the clinical manifestations may be different, and the difficulty and complexity of root canal therapy are different. With the development of medical technology, cluster nursing based on evidence-based medicine has become one of the important nursing models, which takes scientific evidence as the main basis, attaches importance to human factors, and aims at fully understanding and respecting the wishes and needs of different patients. It is the most influential, most worthy of clinical application, and the worthiest of promotion and recognition of an effective measure [23]. Cluster nursing is a collection of measures, so it is systematic and holistic; each measure is based on evidence-based medicine, which is scientific and aimed at a certain problem, having pertinence and purpose, several measures influence and interact with each other, and the effect of coordinated implementation is far greater than that of a certain measure, with effectiveness and cooperation. It has been unanimously recognized by many clinical personnel [24, 25]. As a new evidence-based medicine concept, ERAS is not a new technology or method, but the optimization of existing perioperative management measures [26]. The clinical effect of ERAS regimen in a variety of operations has been verified. A number of randomized controlled trials and case-control studies have confirmed that the application of ERAS regimen in surgery is safe and effective, which can contribute to the functional recovery of patients and shorten postoperative hospital stay and reduce medical expenses [27]. Meanwhile, our current study indicates that, compared with routine nursing, ERAS can be employed in oral outpatients, which can effectively relieve pain and improve negative emotion, indicating that the application of ERAS in oral outpatients is safe and effective.

The scores of comforts and self-efficacy in the research group were higher than those in the control group, the scores of SAS and SDS in the research group were lower than those in the control group, and the scores of VAS and NRS in the study, demonstrating that the concept of ERAS and cluster nursing can effectively relieve pain, reduce negative emotions, and improve patients' comfort, satisfaction, and self-efficacy. Root canal therapy is to remove the infectious substances in the pulp chamber and root canal by root canal preparation, then close the root canal in a three-dimensional space by root canal disinfection and strict root canal filling, cut off the infection pathway, and promote the healing of pulp disease and periapical lesions [28]. There are many causes of root canal pain, such as bacterial factors, iatrogenic factors, the patient's own physique, and the anatomical location of the affected teeth. Under the existing conditions, doctors have to take anesthetic injection to appease and comfort, but it is sometimes difficult to complete the whole course of root canal therapy. The pain feeling of root canal therapy has a certain impact on the patient's body and mind, resulting in the patient not returning to see the doctor on time and refusing to see a doctor when the affected tooth appears again in the oral cavity after seeing a doctor, which threatens the oral health condition and causes trouble to the patient's daily life [28]. In our study, the nursing satisfaction of the research group was higher than that of the control group.

As early as 1930, the theory of happiness was first put forward. Only with happy emotions can we have a healthy body and a harmonious life. Therefore, subjective well-being is used to describe the happiness of patients in this paper. With regard to the concept of subjective well-being (SWB), psychologists have different understandings of it according to their own research results. The overall evaluation of an individual's quality of life is according to the standards set by himself. Subjective well-being has the characteristics of subjectivity, stability, and integrity [29]. Combined with the results of the current study, the scores of life satisfaction, interpersonal harmony, and self-efficacy in the research group were higher than those in the control group, while the scores of physiological function, psychological function, social function, and health self-cognition in the research group were lower than those in the control group. In the research of Chinese scholars [30], words such as happiness, overall well-being, well-being, subjective quality of life, and happy life index are also utilized to express the concept of subjective well-being. Some studies have pointed out that SWB is an important attitude towards life, which can not only reflect the level of mental health but also measure the quality of life and psychological development. Through the employment of the concept of ERAS and cluster nursing, we could effectively improve the SWB of oral outpatients with root canal therapy and further improve the quality of life. There are some limitations in this study. First, the sample size of this study is not large and it is a single-center study, so bias is inevitable. In future research, we will carry out multicenter, large-sample prospective studies, or more valuable conclusions can be drawn.

Collectively, the adoption of the concept of ERAS and cluster nursing can effectively improve the psychological state and pain score of oral outpatients undergoing root canal therapy, improve comfort and self-efficacy, and enhance subjective well-being and quality of life. ERAS and cluster nursing is of great significance in relieving pain after root canal therapy in outpatient department, reducing patients' pain, and improving patients' quality of life.

## Figures and Tables

**Figure 1:** Nursing satisfaction between the two groups.

**Table 1:** Comfort and self-efficacy scores ($\bar{x}\pm s$, points).

Grouping	Cases	Comfort degree		Self-efficacy	
		Before nursing	After nursing	Before nursing	After nursing
Control group	100	58.53 ± 3.42	76.81 ± 2.45^a^	16.43 ± 2.69	26.48 ± 2.87^a^
Research group	100	58.68 ± 3.64	84.52 ± 2.53^b^	16.96 ± 2.86	36.81 ± 1.46^b^
*t* value		0.300	21.891	1.349	32.080
*P* value		0.764	*P* ≤ 0.001	0.178	*P* ≤ 0.001

Note: the control group before and after nursing, ^a^*P* < 0.05; the research group before and after nursing, ^b^*P* < 0.05.

**Table 2:** The subjective well-being scores ($\bar{x}\pm s$, points).

Grouping	Cases	Before nursing			After nursing		
		Life satisfaction	Interpersonal harmony	Sense of efficacy	Life satisfaction	Interpersonal harmony	Sense of efficacy
Control group	100	25.95 ± 3.91	29.73 ± 2.32	40.75 ± 3.91	30.86 ± 3.95	34.91 ± 3.85	43.91 ± 2.55
Research group	100	25.82 ± 3.44	29.85 ± 2.91	40.81 ± 3.56	35.79 ± 3.11	38.96 ± 3.81	48.96 ± 3.91
*t* value		0.249	0.322	0.322	9.806	7.477	10.818
*P* value		0.803	0.747	0.747	*P* ≤ 0.001	*P* ≤ 0.001	*P* ≤ 0.001

**Table 3:** SAS and SDS scores between the two groups ($\bar{x}\pm s$, points).

Grouping	Cases	SAS		SDS	
		Before nursing	After nursing	Before nursing	After nursing
Control group	100	56.91 ± 3.42	43.66 ± 1.64^a^	59.67 ± 1.53	47.71 ± 1.81^a^
Research group	100	56.31 ± 3.43	38.42 ± 1.11^b^	59.31 ± 1.12	39.43 ± 1.64^b^
*t* value		0.113	26.460	1.898	33.899
*P* value		0.909	*P* ≤ 0.001	0.059	0.031

Note: the control group before and after nursing, ^a^*P* < 0.05; the research group before and after nursing, ^b^*P* < 0.05.

**Table 4:** VAS and NRS scores ($\bar{x}\pm s$, points).

Grouping	Cases	VAS		NRS	
		Before nursing	After nursing	Before nursing	After nursing
Control group	100	4.63 ± 0.89	3.76 ± 0.53^a^	4.88 ± 1.22	3.42 ± 0.57^a^
Research group	100	4.65 ± 0.81	2.44 ± 0.87^b^	4.91 ± 1.27	2.06 ± 0.56^b^
*t* value		0.166	12.957	0.170	17.019
*P* value		0.868	*P* ≤ 0.001	0.864	0.031

Note: the control group before and after nursing, ^a^*P* < 0.05; the research group before and after nursing, ^b^*P* < 0.05.

**Table 5:** Quality of life scores before nursing ($\bar{x}\pm s$, points).

Grouping	Cases	Physiological function		Psychological function		Social function		Healthy self-cognition	
		Before nursing	After nursing	Before nursing	After nursing	Before nursing	After nursing	Before nursing	After nursing
Control group	100	15.68 ± 4.56	13.96 ± 2.13^a^	16.81 ± 3.58	14.66 ± 4.32^a^	18.65 ± 3.52	16.53 ± 2.12^a^	15.64 ± 3.56	13.12 ± 1.34^a^
Research group	100	15.53 ± 4.51	10.56 ± 2.53^b^	16.95 ± 3.92	10.56 ± 1.21^b^	18.42 ± 3.23	10.68 ± 3.66^b^	15.53 ± 3.67	10.45 ± 2.42^b^
*t* value		0.233	10.280	0.263	9.139	0.481	13.830	0.215	9.652
*P* value		0.815	*P* ≤ 0.001	0.792	*P* ≤ 0.001	0.630	*P* ≤ 0.001	0.829	*P* ≤ 0.001

## Data Availability

No data were used to support this study.
